# Efficient Encapsulation of Citral in Fast-Dissolving Polymer-Free Electrospun Nanofibers of Cyclodextrin Inclusion Complexes: High Thermal Stability, Longer Shelf-Life, and Enhanced Water Solubility of Citral

**DOI:** 10.3390/nano8100793

**Published:** 2018-10-06

**Authors:** Zeynep Aytac, Asli Celebioglu, Zehra Irem Yildiz, Tamer Uyar

**Affiliations:** Institute of Materials Science & Nanotechnology, UNAM-National Nanotechnology Research Center, Bilkent University, Ankara 06800, Turkey; zynpytc@gmail.com (Z.A.); aslicelebi06@gmail.com (A.C.); zehra.gurbuz@bilkent.edu.tr (Z.I.Y.)

**Keywords:** cyclodextrin, electrospinning, nanofiber, inclusion complex, citral, enhanced water solubility, high thermal stability, longer shelf-life

## Abstract

Here, we report a facile production of citral/cyclodextrin (CD) inclusion complex (IC) nanofibers (NFs) from three types of CDs (hydroxypropyl-beta-cyclodextrin (HPβCD), hydroxypropyl-gamma-cyclodextrin (HPγCD), and methylated-beta-cyclodextrin (MβCD)) by an electrospinning technique without the need of any polymeric carrier matrix. Self-standing nanofibrous webs of citral/CD-IC nanofibers (citral/CD-IC-NF) with uniform fiber morphology have been successfully electrospun from aqueous solutions of citral/CD-IC. Thanks to the inclusion complex formed with CDs, the efficient preservation of citral (up to ~80%) in citral/CD-IC-NFs was observed. In addition, the citral/CD-IC-NFs have shown ~50% preservation of citral for 15 days at room temperature even though citral has a highly volatile nature. The enhanced thermal stability of citral (~100–300°C) in citral/CD-IC-NFs compared to pure citral (~50–165°C) has been observed. Moreover, citral/CD-IC-NFs tended to disintegrate in water very quickly. To summarize, citral was efficiently encapsulated in citral/CD-IC-NFs, and these citral/CD-IC-NFs have been shown to be fast dissolving. In citral/CD-IC-NFs, citral/CD-ICs have enhanced water solubility of citral along with high-temperature stability and a longer shelf-life.

## 1. Introduction

Citral (3,7-dimethyl-2,6-octadienal) is a flavor/fragrance molecule found in lemongrass oil that possesses a lemon-like odor and a bittersweet taste (Figure 1). Citral is composed of two geometric isomers, geranial and neral, which have an intense lemon odor and a sweet taste, respectively. However, citral has low aqueous solubility and is unstable against heat, air, and light [1]. Cyclodextrins (CDs) (Figure 1) hold exceptional complexation capability due to the relatively hydrophobic cavity of the interior of these supramolecular structures and offer an excellent feature to encapsulate a variety of compounds that have appropriate polarity and dimensions that fit into the CD cavity. Similar to other encapsulating methods, the inclusion complexation with CDs provides many advantages to the guest molecules, including enhanced water solubility, higher thermal stability, a longer shelf-life, etc. There are different native CDs and chemically modified CDs (Figure 1a) available on the market that can be used to design appropriate CD-IC systems for different guest molecules [2,3,4]. Modified CDs are considered an important class of CDs owing to their higher water solubility compared to native CDs. This feature is also important for achieving nanofibers via electrospinning from highly concentrated aqueous solutions of modified CDs [5,6,7]. Thus, CD-IC nanofibers have been produced from CD-IC systems of an antibacterial triclosan [8,9] and flavors/fragrances such as geraniol [10], vanillin [11], limonene [12], linalool [13], cineole and p-cymene [14], camphor [15], and an antioxidant vitamin E [16] from our previous studies. 

Citral is a clear yellow liquid that is highly volatile and not very soluble in water. However, the inclusion complexation of citral with cyclodextrin could provide higher stability at high temperatures and enhanced water solubility. Citral is a common and widely used compound as a flavor/fragrance and bactericide in food and medical applications. Therefore, encapsulation of citral in a nanofiber matrix may be quite applicable in the food and medical fields. In this study, we aimed to achieve higher thermal stability, enhanced water solubility, and a longer shelf-life for citral through forming a citral/cyclodextrin inclusion complex (citral/CD-IC) and to transform citral/CD-IC into self-standing solid-state nanofibrous webs by electrospinning.

Electrospinning is a well-known technique for producing nanofibers from various materials. Polymers are the materials of choice for producing nanofibers by electrospinning due to their fiber forming property [17,18,19]. Moreover, electrospinning active additive-loaded polymeric nanofibers yields functional polymeric nanofibers in one step [20]. Therefore, CD-ICs of volatile active agents can also be loaded in polymeric nanofibers to control the release of active agents by maintaining their chemical/biological activities [21,22]. Besides, polymer-free CD-IC nanofibers could be an alternative to polymeric nanofibers into which CD-ICs are incorporated, since CD-IC incorporated polymeric nanofibers have drawbacks, such as the use of organic solvents during the production of CD-IC incorporated polymeric nanofibers and sometimes only limited amounts of active agents can be loaded into the fiber matrix [8,9,10,11,12,13,14,15,16].

The literature studies on citral/CD-inclusion complexes are mostly related to the powder form of citral/CD-ICs [1,23,24]. In these reports, the inclusion complexes of citral and different CD types (α-CD, β-CD, γ-CD, hydroxypropyl-β-CD, and monochlorotriazinyl-β-CD) were formed in the powder form, and the interactions in CD-IC were comparatively studied. As a totally new approach for citral/CD-IC systems, in the present study, citral/CD-ICs (Figure 1b) were obtained first with three types of CDs—(hydroxypropyl-β-cyclodextrin (HPβCD), hydroxypropyl-γ-cyclodextrin (HPγCD), and methylated-β-cyclodextrin (MβCD)) (Figure 1a)—in highly concentrated aqueous solution, and then nanofibers (citral/CD-IC-NF) in the form of self-standing webs were produced from the aqueous solutions of these citral/CD-ICs via electrospinning (Figure 1c). The highly concentrated citral/CD-IC solutions enabled the electrospinning of citral/CD-IC-NFs without the need of a polymeric carrier matrix [5,6]. In addition, CD-ICs offer advantages, including enhanced water solubility and high thermal stability and a longer shelf-life for the hydrophobic and volatile guest molecules. Here, the water solubility of the citral/CD-IC systems was analyzed by a phase solubility diagram. The fiber morphology of citral/CD-IC-NF, which is bead-free and uniform, was confirmed by scanning electron microscopy (SEM) imaging. Nuclear magnetic resonance (^1^H NMR) was used to calculate the molar ratios of CDs and citral in citral/CD-IC-NF. Further, the CD-IC formation was analyzed by X-ray diffraction (XRD) and Fourier-transform infrared spectrophotometer (FTIR) studies. The thermal stabilities of citral/CD-IC-NFs were evaluated using thermal gravimetric analysis (TGA). Photographs of the citral/CD-IC-NFs were also taken to show the self-standing characteristic of these nanofibrous materials. The fast-dissolving nature of the citral/CD-IC-NFs was recorded and compared to citral/CD-IC in powder form.

## 2. Materials and Methods 

### 2.1. Materials

Hydroxypropyl-beta-cyclodextrin (HPβCD, degree of substitution: ~0.6, Cavasol^®^W7 HP Pharma), hydroxypropyl-gamma-cyclodextrin (HPγCD, degree of substitution: ~0.6, Cavasol^®^W8 HP Pharma), and methylated-β-cyclodextrin (MβCD, degree of substitution: 1.6–1.9, Cavasol^®^W7 M Pharma) were kindly donated by Wacker Chemie (Munich, Germany). Citral (≥95%, Sigma Aldrich, Hamburg, Germany), deuterated dimethylsulfoxide (DMSO-d6, deuteration degree min 99.8% for ^1^H NMR spectroscopy, Merck, Germany), potassium bromide (KBr, 99%, FTIR grade, Sigma-Aldrich, Germany), and poly(vinyl alcohol) (PVA, Mw 85000–124000 g/mol, Sigma Aldrich, 87%–89% hydrolysed, Germany) were purchased. Above-mentioned materials were used as-received without any modification. A Millipore Milli-Q ultrapure water system was used to obtain distilled-deionized water that was used for the experiments.

### 2.2. Preparation of the Citral/CD-IC

Inclusion complexes (ICs) of cyclodextrins (CDs) (HPβCD, HPγCD, and MβCD) with citral were synthesized by dissolving 160% (w/v) CDs in aqueous solutions and then adding citral equivalent to a 1:1 molar ratio to those CD solutions. Initially, the citral/CD-IC solutions were turbid but later became clear and homogenous with the dissolution of citral over the time. The solutions were kept by stirring them at room temperature (RT) for 12 h in tightly sealed glass vials. Then, electrospinning was performed. The composition of the solutions, the viscosity and conductivity measured from the solutions, the morphological characteristics of citral/CD-IC nanofibers (citral/CD-IC-NFs), and the average fiber diameter (AFD) of citral/CD-IC-NFs are shown in Table 1. Pure CD nanofibers without citral (HPβCD-NF, HPγCD-NF, and MβCD-NF) were also prepared according to our previous reports and used as reference samples [5,6]. Thus, we have managed to produce nanofibers from 160% (w/v) of HPβCD, 140–160% (w/v) of MβCD, and 160% (w/v) of HPγCD solutions. The powder form of citral/CD-ICs was also synthesized using the freeze-drying technique for a comparative study. Initially, 160% (w/v with respect to solution) CD (HPβCD, HPγCD, and MβCD) was dissolved in water. Afterward, the required amount of citral was added to the solutions to give a 1:1 molar ratio. Then, the solutions were freeze-dried (Labconco, Corporation, Kansas City, MO, USA). 

### 2.3. Electrospinning 

To produce citral/CD-IC-NFs, each citral/CD-IC solution (citral/HPβCD-IC, citral/HPγCD-IC and citral/MβCD-IC) was separately loaded in syringes having a metallic needle of 0.4 mm inner diameter. Then, the syringe pump (KD Scientific, KDS-101, Holliston, MA, USA) was put on and pumped at a rate of 0.5 mL/h toward the collector covered with a piece of aluminum foil. The distance and electric field applied to the system (AU Series, Matsusada Precision Inc., Osaka, Japan) was arranged as 10–15 cm and 15–20 kV, respectively. The electrospinning was carried out in an enclosed Plexiglas box at 25°C and 18% relative humidity. The electrospun webs of citral/CD-IC-NFs were kept in a refrigerator (4°C) prior to analysis. For a comparative time-dependent stability study, a polymeric system without CD-IC was also tested. That is, PVA (10% w/v with respect to solvent) nanofibers with only citral (10% w/w with respect to polymer) (citral/PVA-NF)) were also produced from citral/PVA aqueous solution by electrospinning.

### 2.4. Measurements and Characterization

To determine the solubility enhancement of citral by complexation with CDs, phase solubility measurements were performed for citral/CD-IC systems based on the method improved by Higuchi and Connors [25]. Thus, suspensions were obtained by adding excess amounts of citral to CD (HPβCD, HPγCD, and MβCD) solutions that were prepared in water (10 mL) and they were stirred at RT for 48 h. Then, a membrane filter (0.45 µm) was used to filter the resulting suspensions. After the filtration, the absorption of the solutions was measured at 243 nm by UV spectroscopy (Varian, Cary 100). The phase solubility experiments were repeated three times. The solubility results are given as the average ± standard deviation by calculating the average and standard deviation.

The stability constant (K_S_) of each system was calculated from the equation provided below:

K_S_=slope/S_0_ (1−slope) (1)

where S_0_ is the intrinsic solubility of citral (3.8 mM) when there is no CD [26].

The viscosity of each citral/CD-IC solution prepared with three different CD types was measured at RT via Anton Paar Physica MCR 301 (Graz, Austria) rheometer with a spindle of CP 20-4 at a shear rate of 100 s^−1^. The conductivity of the solutions was also measured at RT using Inolab^®^ pH/Cond 720-WTW (Jakarta, Indonesia).

Scanning electron microscopy (SEM, FEI - Quanta 200 FEG, Hillsboro, OR, USA) was used to capture the images for each nanofiber achieved and the morphology and average fiber diameter (AFD) (*n* ≥ 100) of the nanofibers were determined based on the SEM images. Nanofiber samples were sputtered with 5 nm of Au/Pd (PECS-682, Pleasanton, CA, USA) to minimize charging of the samples during SEM imaging. 

Then, 5 mL of water was added to the citral/CD-IC-NF and citral/CD-IC powders in Petri dishes and videos were recorded to show the water solubility character of each sample. For a visual comparison, pure citral (equivalent to the amount in the nanofibers) was dropped into 5 mL of aqueous solution. 

To decide the molar ratio of CDs to citral by ^1^H NMR (Bruker DPX-400, Mannheim, Germany), 10 mg of citral/CD-IC-NFs and citral/polyvinyl alcohol-nanofibers (citral/PVA-NF) were dissolved in 500 µL of d6-dimethyl sulfoxide (d6-DMSO). The characteristic chemical shifts (δ, ppm) of each compound were determined and the integration of each peak was determined using Mestrenova software. Finally, the molar ratio of CD and citral in citral/CD-IC-NFs was calculated by the proportion of the integration of the peaks from CD and citral. 

The thermal properties of pure citral, CD-NFs, and citral/CD-IC-NF were studied by thermogravimetric analysis (TGA) (TA Q500, New Castle, DE, USA) under nitrogen atmosphere by heating the samples at a heating rate of 20 °C/min from 25°C to 500°C. Contrary to other samples, citral was heated to 200°C due to its volatile nature. 

To check the time-dependent release profile of the samples, citral/CD-IC-NF and citral/PVA-NF were kept in the open air in the laboratory for 15 days (RT, 18% RH). ^1^H NMR measurements were performed at definite time intervals to determine the amount of citral remaining in the nanofibers.

X-ray diffraction (XRD) (PANalytical X’Pert powder diffractometer, Texas, USA) was employed to characterize the crystalline structure of CD-NF and citral/CD-IC-NF from 2θ = 5° to 30° using Cu Kα radiation in powder diffraction configuration. XRD analysis could not be performed for pure citral because of the liquid state of citral at RT.

The potassium bromide (KBr) pellets were prepared to obtain infrared spectra of the samples by mixing samples with KBr before the measurement. Then, the infrared spectra of citral, CD-NF, and citral/CD-IC-NFs were obtained in the range of 4000 cm^−1^ and 400 cm^−1^ via Fourier-transform infrared spectrophotometer (FTIR) (Bruker-VERTEX 70, Mannheim, Germany). The parameters for the measurements were decided as 64 scans and a resolution of 4 cm^−1^.

## 3. Results and Discussion

### 3.1. Phase Solubility Studies

The linear increment in the solubility of citral with increasing concentrations of CDs regardless of the CD type in phase solubility diagrams of citral/CD systems indicate that the diagrams are linear (A_L_) type, which demonstrates that the complexes formed in a 1:1 molar ratio (Figure 2) [27]. In a similar study on citral, Okada et al. [28] suggested that the solubility of citral was improved with a different type of β-CD. Moreover, Phunpee et al. [1] investigated the phase solubility change of citral with three native CD types and revealed that the solubility of citral was enhanced because of complex formation. In our study, the stability constant (K_S_) values of the complexes were calculated based on Equation 1. The K_S_ values of citral/HPβCD-IC, citral/HPγCD-IC, and citral/MβCD-IC were determined as 505 M^−1^, 219 M^−1^, and 1375 M^−1^, respectively. K_S_ values essentially represent the binding strength between the guest molecules and CD and, based on our results, the stabilities of the complexes were in the order of MβCD > HPβCD > HPγCD. Here, the bigger cavity size of HPγCD prevented it from being as efficient as HPβCD and MβCD in stabilizing the interactions with citral in the dynamic environment of the system. On the other hand, the MβCD-based system (1375 M^−1^) indicates a higher stability constant than HPβCD system (505 M^−1^). Here, the less polar feature of MβCD compared to HPβCD might be influential for the more stable complexation between the hydrophobic citral molecules and MβCD in the polar water environment [29].

### 3.2. Morphology Analyses of Nanofibers 

SEM images and the photographs of citral/HPβCD-IC nanofibers (citral/HPβCD-IC-NF), citral/HPγCD-IC nanofibers (citral/HPγCD-IC-NF), and citral/MβCD-IC nanofibers (citral/MβCD-IC-NF) webs are given in Figure 3. The production of uniform and bead-free nanofibers was confirmed by SEM imaging of citral/HPβCD-IC-NF, citral/HPγCD-IC-NF, and citral/MβCD-IC-NF. Additionally, electrospun polymeric citral/PVA-NF, which has 185 ± 30 nm of average fiber diameter, was also obtained with bead-free and uniform fiber morphology (Figure S1). As we reported in our previous studies [5,6], CDs are capable of forming self-assemblies and aggregations in the highly concentrated CD solutions, which help the electrospinnability and fiber formation during electrospinning. Even though citral/CD-IC is a non-polymeric system consisting of small molecules, self-standing and flexible nanofibrous materials were obtained from citral/CD-IC-NFs (Figure 3d–f). 

The average fiber diameters (AFD) of citral/HPβCD-IC-NF (105 ± 35 nm), citral/HPγCD-IC-NF (1380 ± 380 nm), and citral/MβCD-IC-NF (125 ± 35 nm) were measured from SEM images. The ultimate fiber morphology and fiber diameter are affected by various electrospinning parameters and the distance between the needle and collector is one of them. This parameter has been examined and reported by different studies in the literature, and the main observation is that the increasing distance between collector and needle leads to thinner fiber formation due to the longer exposure time of stretching of the electrospun fibers [30,31,32]. In our study, we first aimed to obtain bead-free and uniform fibers from citral/CD-IC, and so we optimized our system at the given range of collection distance (10–15 cm). During our optimization study, definite fiber diameter differences were not observed for citral/CD-IC solutions depending on the collector needle distance within 10–15 cm. However, the viscosity and conductivity differences of the citral/CD-IC solutions were the main reasons for the variation in the AFD of citral/CD-IC-NF samples (Table 1). Since the solvent type has a significant influence on the viscosity and conductivity of electrospinning solutions, it is a more dominant parameter for the morphology of the resulting electrospun fibers [5,6,11,19,33]. In one of our previous studies, the electrospinning of vanillin/CD-IC was investigated in three different solvent types (DMSO, dimethylformamide (DMF), and water) [11]. The results of the study indicated that it is possible to get fibers from less concentrated CD solutions prepared in DMF and DMSO compared to a water system. However, thicker fiber diameters were obtained from organic solvent-based electrospinning of CD-ICs when compared to a water-based CD-IC system. More importantly, the use of organic solvents creates toxicity problems for food-related applications of these CD-IC electrospun fibers. Therefore, water was chosen as a solvent system in this study to support food-related applications of citral/CD-IC-NF samples. Solutions having low viscosity and high conductivity yield thinner fibers owing to the increased jet stretching in electrospinning [33]. In our case, the lower conductivity and higher viscosity of citral/HPγCD-IC solutions caused citral/HPγCD-IC-NF to obtain a much higher AFD (1380 ± 380 nm) compared to citral/HPβCD-IC-NF (105 ± 35 nm) and citral/MβCD-IC-NF (125 ± 35 nm), because the electrospinning of the citral/HPγCD-IC system was subjected to less stretching during the electrospinning process. On the other hand, both citral/HPβCD-IC and citral/MβCD-IC solutions had lower viscosity and higher conductivity values resulting in a much smaller AFD; citral/HPβCD-IC-NF had an AFD of 105 ± 35 nm and citral/MβCD-IC-NF had an AFD of 125 ± 35 nm. 

Furthermore, the visual water solubility test was performed for pure citral and citral/CD-IC-NF webs. A volume of 5 mL of water was added to the citral/CD-IC-NF web samples (Video S1) and pure citral (approximate amount of citral in the nanofibers) was dropped into 5 mL of water (Video S2) for a comparative study. As seen in the Videos S1–S2 and Figure 4, citral could not be dissolved in water. However, rapid disintegration and dissolution of citral/CD-IC-NF webs occurred within a very short time period (in a second or so). The comparative solubility test of freeze-dried citral/CD-IC (powder) was performed as well. It was observed that citral/CD-IC-NF webs could disintegrate more readily in water than citral/CD-IC (powder) (Video S3) due to the high surface area and nanoporous structures of the nanofibrous webs, facilitating the penetration and ultimately interaction of water molecules within the web samples.

### 3.3. The Molar Ratio of Citral/CD-IC

The molar ratios of citral:CD in citral/CD-IC-NF samples were calculated by taking the integration of the protons of citral and CD from ^1^H NMR spectra of citral/HPβCD-IC-NF, citral/HPγCD-IC-NF, and citral/MβCD-IC-NF (Figure 5 and Figure S2). Here, ^1^H NMR measurements were performed after the electrospinning process by dissolving citral/CD-IC-NF samples in d6-DMSO. The molar ratios of citral:HPβCD, citral:HPγCD, and citral:MβCD were found as ~0.60:1.00, ~0.60:1.00, and ~0.80:1.00 for citral/HPβCD-IC-NF, citral/HPγCD-IC-NF, and citral/MβCD-IC-NF, respectively. The amount of citral protected from evaporation calculated from ^1^H NMR spectra is in agreement with the calculated amount of citral from TGA results recorded concurrently to ^1^H NMR measurements, which will be discussed in the following section.

The time-dependent stability (up to 15 days) of citral in citral/CD-IC-NF samples was evaluated by ^1^H NMR measurements, and the results are summarized in Table S1. To show the effect of cyclodextrin inclusion complexation, the polymeric electrospun nanofiber matrix without CD-IC (citral/PVA-NF sample) was also tested as a comparative study. After electrospinning (t = 0 day, the storage time is less than 3 h), the molar ratios of citral:HPβCD, citral:HPγCD, and citral:MβCD were calculated from ^1^H NMR (0th day in Table S1) as ~0.65:1.00, ~0.60:1.00, and ~0.85:1.00 for citral/HPβCD-IC-NF, citral/HPγCD-IC-NF, and citral/MβCD-IC-NF, respectively. After 15 days of storing at room temperature, the molar ratios of citral:HPβCD, citral:HPγCD, and citral:MβCD were ~0.50:1.00, ~0.40:1.00, and ~0.45:1.00 for citral/HPβCD-IC-NF, citral/HPγCD-IC-NF, and citral/MβCD-IC-NF, respectively. Although citral has a volatile nature, our results showed that the release of citral from citral/CD-IC-NF during the storage at room temperature was minimal. Citral/HPγCD-IC-NF had the least amount of citral in the beginning and it showed slightly lower preservation efficiency in total, which is most likely because it had the lowest K_S_, calculated from phase solubility diagrams. The lower strength of the interaction with HPγCD might be related to the bigger cavity size of this CD type as compared to β-CD derivatives. In conclusion, β-CD derivatives were able to keep more citral in the nanofibers than HPγCD. Here, citral/PVA-NF without CD-IC was also electrospun for the comparative study to examine the effect of inclusion complexation on the stability of citral in the fiber matrix during and after electrospinning. PVA polymer was chosen because it is comparable to CD based on its electrospinnability in water and its possession of hydroxyl moieties in its structure. The presence and the time-dependent stability of citral in citral/PVA-NF were also studied after electrospinning and storing the sample at RT for up to 15 days (Figure S3). However, the related peaks of citral could not be observed in the ^1^H NMR spectrum of the citral/PVA-NF sample, which was tested just after the electrospinning (Figure S3). The results reveal that citral/PVA-NF could not preserve citral during either the electrospinning process or the short time storage just after electrospinning. On the contrary, a significant amount of citral (up to ~50%) was preserved in citral/CD-IC-NF webs even after 15 days of storage at RT. Therefore, it can be concluded that inclusion complexation provides time-dependent stability for volatile compounds in CD-IC-NFs compared to the polymeric nanofibrous matrix without CD-IC.

### 3.4. Thermal Analysis of Nanofibers

The TGA was used to investigate the thermal stability of citral/HPβCD-IC-NF, citral/HPγCD-IC-NF, and citral/MβCD-IC-NF webs (Figure 6). The TGA of pure citral and pure CD-NF samples was also carried out for comparison. HPβCD-NF, HPγCD-NF, and MβCD-NF exhibited a weight loss of water below 100 °C and the main thermal degradation of CD was above 275 °C. Citral is a volatile compound and evaporates between the temperature of 50 °C and 165 °C. The volatility of citral was reduced when it was inserted in the CD cavity. Thus, the evaporation of citral increased to a much higher temperature in citral/HPβCD-IC-NF (100–255 °C), citral/HPγCD-IC-NF (100–270 °C), and citral/MβCD-IC-NF (80–185 °C and 260–305 °C). Therefore, it was concluded that complexation was formed between CDs and citral. Other researchers also reported an improvement in citral’s thermal stability when complexation is formed with CDs [23,34]. The citral/HPβCD-IC-NF has a three-step weight loss; below 100 °C, at 100–255 °C, and at 255–415 °C, which is attributed to water loss, evaporation of citral, and the main thermal degradation of HPβCD, respectively. Accordingly, the amount of citral remaining in the nanofibers was calculated as 5.96% (w/w) in citral/HPβCD-IC-NF. Similarly, a three-step weight loss was observed in citral/HPγCD-IC-NF: below 100 °C, at 100–270 °C, and at 270–410 °C, which was attributed to the loss of water molecules, evaporation of citral, and HPγCD’s main thermal degradation, respectively. From this result, the amount of citral was determined as 5.33 % (w/w) in citral/HPγCD-IC-NF. Unlike citral/HPβCD-IC-NF and citral/HPγCD-IC-NF, citral/MβCD-IC-NF exhibited a four-step weight loss. The first weight loss below 100 °C was due to the water loss and the final weight loss that occurred between 305 °C and 420 °C corresponds to the main thermal degradation of MβCD. The second and the third weight losses observed at 80–185 °C and 260–305 °C in citral/MβCD-IC-NF might be due to the presence of two types of complexes that have interactions of different strengths. Thus, the total amount of citral in citral/MβCD-IC-NF was calculated as 9.16% (w/w) (6.32% (w/w) from the first weight loss and 2.84% (w/w) from the second weight loss. To summarize, up to ~65% of citral was preserved in citral/HPβCD-IC-NF and citral/HPγCD-IC-NF, whereas ~93% of citral was preserved in citral/MβCD-IC-NF. The molar ratios of citral:HPβCD, citral:HPγCD, and citral:MβCD were calculated as ~0.65:1.00, ~0.65:1.00, and ~0.90:1.00 from TGA results in citral/HPβCD-IC-NF, citral/HPγCD-IC-NF, and citral/MβCD-IC-NF, respectively. The results show that the molar ratio of citral:CD in citral/CD-IC-NF samples calculated from TGA correlates with the results obtained from ^1^H NMR. According to ^1^H NMR and TGA data, it was concluded that MβCD can provide better encapsulation of citral. These results correlate with the phase solubility studies in which a higher K_S_ value and a stronger interaction between citral and MβCD was observed. 

Furthermore, because the water molecules in the cavity of CDs were replaced with guest molecules during the complex formation, a reduction of water is expected when a guest molecule is complexed within the cavity of CDs. The amount of water calculated from the water loss below 100 °C in TGA graphs of pure HPβCD-NF, HPγCD-NF, and MβCD-NF was 4.83%, 5.80%, and 2.45% (w/w), respectively (Figure 6). The amount of water decreased to 1.15%, 1.10%, and 1.40% (w/w) for citral/HPβCD-IC-NF, citral/HPγCD-IC-NF, and citral/MβCD-IC-NF, respectively. The reduction in the water content in the citral/CD-IC-NF samples strongly suggests complex formation between with three CD types and citral in these webs. 

### 3.5. Structural Characterization of Nanofibers

Structural characterization of citral/HPβCD-IC-NF, citral/HPγCD-IC-NF, and citral/MβCD-IC-NF was performed by using XRD and FTIR. XRD patterns of HPβCD-NF, HPγCD-NF, MβCD-NF, citral/HPβCD-IC-NF, citral/HPγCD-IC-NF, and citral/MβCD-IC-NF are given in Figure 7a. Citral/HPβCD-IC-NF, citral/HPγCD-IC-NF, and citral/MβCD-IC-NF exhibited an amorphous pattern similar to pure HPβCD-NF, HPγCD-NF, and MβCD-NF. XRD data for pure citral could not be recorded since it is in a liquid state at RT; even so, citral/CD-IC-NF also had an amorphous structure. In addition, there was no crystal formation of citral in citral/CD-IC-NF, suggesting that there was an inclusion complexation between the two compounds used (Figure 7a).

FTIR analyses of citral, HPβCD-NF, HPγCD-NF, MβCD-NF, citral/HPβCD-IC-NF, citral/HPγCD-IC-NF, and citral/MβCD-IC-NF are presented in Figure 7b,c. CDs exhibited characteristic absorption peaks at around 1030 cm^−1^ (coupled C–C stretching vibration), 1080 cm^−1^ (coupled stretching C–O vibration), 1157 cm^−1^ (antisymmetric stretching vibration of C–O–C glycosidic bridge), 1638 cm^−1^ (H–OH bending), 2925 cm^−1^ (C–H stretching), and 3401 cm^−1^ (O–H stretching) [10,12]. The characteristic peaks of citral appeared at 1380 cm^−1^ of bending (CH_3_) vibration, 1443 cm^−1^ of C=C vibration, 1674 cm^−1^ of C=O stretching vibration, and 2847 cm^−1^ and 2916 cm^−1^ of CH_2_ and CH_3_ stretching vibration [23]. Because the characteristic peaks of CDs at 2925 cm^-1^ and 1638 cm^−1^ and citral at 2916 cm^−1^, 2847 cm^−1^, and 1674 cm^−1^ overlap, it is difficult to differentiate them. However, the peaks of CDs are observed at 1036 cm^1^, 1083 cm^−1^, and 1155 cm^−1^ for citral/HPβCD-IC-NF, 1031 cm^−1^, 1082 cm^−1^, and 1155 cm^−1^ for citral/HPγCD-IC-NF, and 1043 cm^−1^, 1089 cm^−1^, and 1171 cm^−1^ for citral/MβCD-IC-NF (Figure 7c). The shifts of the peaks of CDs indicate the presence of an interaction between CDs and citral. Similarly, Zhu et al. [23] demonstrated that the disappearance or shifting in the peaks at 2966 cm^-1^, 2916 cm^−1^, 2860 cm^−1^, 2759 cm^−1^, and 1674 cm^−1^ might be attributed to complex formation between citral and CDs. The reported shifts seen in the FTIR spectra of CD-ICs compared to pure CDs and citral were regarded as inclusion complexation of citral with the CDs [23,34].

## 4. Conclusions

The flexible and self-standing citral/CD-IC-NF webs were successfully produced using three types of CDs (HPβCD, HPγCD, and MβCD) by an electrospinning technique without any polymeric carrier matrix. Even though citral is quite a volatile molecule, efficient preservation of citral and a longer shelf-life were successfully achieved for citral/CD-IC-NF samples due to inclusion complexation with CD. In addition, citral/CD-IC-NF have shown much higher thermal stability for citral when compared to pure citral. The citral/CD-IC-NF webs had a fast-dissolving character compared to the powder form of citral/CD-IC. Moreover, the water solubility of citral was enhanced for citral/CD-IC-NF. To conclude, citral/CD-IC-NF can be easily utilized and provides advantages for food or related bio applications due to the non-toxic nature of CD and the flavor/fragrance properties of citral.

## Figures and Tables

**Figure 1:** (**a**) The chemical structure of HPβCD, HPγCD, and MβCD, (**b**) the chemical structure of citral and the schematic representation of citral/cyclodextrin (CD) and citral/CD-IC, (**c**) the schematic representation of electrospinning of nanofibers from a citral/CD-IC solution.

**Figure 2:** Phase solubility diagram of (**a**) citral/HPβCD, (**b**) citral/HPγCD, and (**c**) citral/MβCD systems in water (*n* = 3).

**Figure 3:** Scanning electron microscopy (SEM) images of electrospun nanofibers of (**a**) citral/HPβCD-IC NF, (**b**) citral/HPγCD-IC NF, and (**c**) citral/MβCD-IC NF; the photographs of (**d**) citral/HPβCD-IC-NF, (**e**) citral/HPγCD-IC-NF, and (**f**) citral/MβCD-IC-NF webs.

**Figure 4:** Presentation of the solubility behavior of pure citral and citral/HPβCD-IC-NF, citral/HPγCD-IC-NF, and citral/MβCD-IC-NF webs in water (the images were captured from the Videos S1–S2).

**Figure 5:** ^1^H NMR spectra of (**a**) citral/HPβCD-IC-NF, (**b**) citral/HPγCD-IC-NF, and (**c**) citral/MβCD-IC-NF dissolved in d6-DMSO.

**Figure 6:** Thermogravimetric analysis (TGA) thermograms of (**a**) citral, HPβCD-NF, citral/HPβCD-IC-NF, (**b**) citral, HPγCD-NF, citral/HPγCD-IC-NF, and (**c**) citral, MβCD-NF, citral/MβCD-IC-NF.

**Figure 7:** (**a**) X-ray diffraction (XRD) patterns of HPβCD-NF, HPγCD-NF, MβCD-NF, citral/HPβCD-IC-NF, citral/HPγCD-IC-NF, and citral/MβCD-IC-NF; (**b**) full and (**c**) narrow range Fourier-transform infrared (FTIR) spectra of citral, HPβCD-NF, HPγCD-NF, MβCD-NF, citral/HPβCD-IC-NF, citral/HPγCD-IC-NF, and citral/MβCD-IC-NF.

**Table 1:** The properties of the citral/CD-IC (citral/HPβCD-IC, citral/HPγCD-IC, citral/MβCD-IC) solutions used for electrospinning and morphological characteristics of the resulting citral/CD-IC-NF (citral/HPβCD-IC-NF, citral/HPγCD-IC-NF, citral/MβCD-IC-NF) samples.

Solutions	% CD ^a^ (w/v)	% citral ^b^ (w/w)	Viscosity (Pa·s)	Conductivity(μS/cm)	Average Fiber Diameter (AFD) (nm)	Fiber Morphology
Citral/HPβCD-IC-NF	160	9.3	0.27	19.67	105 ± 35	bead-free nanofibers
Citral/HPγCD-IC-NF	160	8.4	0.37	8.26	1380 ± 380	bead-free nanofibers
Citral/MβCD-IC-NF	160	9.9	0.25	15.57	125 ± 35	bead-free nanofibers

^a^ with respect to solvent (water), ^b^ with respect to total weight of the sample.

## Supplementary Materials

The following are available online at http://www.mdpi.com/2079-4991/8/10/793/s1. Figure S1: The representative SEM image of citral/PVA-NF; Figure S2: ^1^H-NMR spectra of (a) HPβCD-NF, (b) HPγCD-NF (c) MβCD-NF, and (d) citral dissolved in d6-DMSO; Figure S3: ^1^H NMR spectra of citral/PVA-NF sample by dissolving citral/PVA-NF in d6-DMSO at certain time intervals. (Time zero means after the electrospinning, the storage time is less than 3 h.); Table S1: The molar ratio of citral:CD in citral/CD-IC-NF samples stored at room temperature for 15 days. (The molar ratio of citral:CD was decided from ^1^H NMR measurements by dissolving citral/CD-IC-NF samples in d6-DMSO at certain time intervals). Video S1: The solubility behavior of citral/CD-IC-NF; Video S2: The solubility behavior of pure citral; Video S3: The solubility behavior of citral/CD-IC powder.
